# Current Status and Factors Associated with Clean Operating Rooms: A Survey of Hospitals in China

**DOI:** 10.1155/2022/8749785

**Published:** 2022-08-12

**Authors:** Ye Lu, Ran Cai, Zhongyi Xie, Xiaodong Gao, Xiaoqiang Huang, Ji Xu, Ye Li, Guoqing Hu

**Affiliations:** ^1^Department of Environmental Health, Zhejiang Provincial Center for Disease Control and Prevention, Hangzhou 310051, China; ^2^Department of Infection Management, Zhongshan Hospital, Shanghai 200032, China; ^3^Department of Infection Management, Xiaolan People' Hospital of Zhongshan, Zhongshan 528400, China

## Abstract

**Background:**

Indoor air quality is controlled in the clean operating room (OR) to reduce the risk of surgical-site infections (SSIs). The aim of this study is to assess the usage and management of clean ORs in China and to identify factors associated with the risk of SSIs.

**Methods:**

An online survey was distributed to hospitals in China from August 5 to September 5, 2018 via the WeChat account of the Shanghai International Forum for Infection Control and Prevention. The questionnaire consisted of two parts: basic information (hospital type, level, and number of beds) and usage and management (number of ORs, usage time, maintenance mode, test frequency, compliance with current standards, and comfort of healthcare workers). The significance of factors associated with the cleanliness and maintenance of clean ORs was assessed by univariate and multivariate logistic regression analyses.

**Results:**

Among 1,308 responding hospitals, 25.7% failed to comply with current standards. “Maintenance mode” had a significant effect on compliance with current standards for clean ORs (*p* < 0.0001) and “professional” maintenance was superior to “outsource or no” maintenance (odds ratio = 0.511, 95% confidence interval = 0.367–0.711). There was a significant difference in the comfort of healthcare workers in clean ORs that complied with current standards vs. those that did not (39.92% [388/972] vs. 64.28% [216/336], respectively, *p* < 0.0001). Humidity was the chief complaint among healthcare workers.

**Conclusion:**

Maintenance of clean ORs was significantly associated with the compliance of current standards. Noncompliance with current standards was associated with greater risks of SSIs. Maintenance of ORs for prevention of SSIs should consider the costs and benefits.

## 1. Introduction

Surgical-site infections (SSIs) are the second most common cause of nosocomial infections worldwide and often result in prolonged hospitalization, increased mortality, and greater medical costs. SSIs account for ∼20% of all nosocomial infections and are associated with a 2–11-fold greater risk of mortality [1–4].

In developed countries, SSI rates reportedly range from 1.2% to 5.2% with even higher rates in developing countries of 5% to 20% [5–8]. A 2019 report by the European Center for Disease Prevention and Control noted that the risk of SSIs ranged from 0.5% to 10.1%, depending on the surgical procedure [9]. Exposure of surgical wounds to airborne microorganisms is a major cause of SSIs. During surgery, air in the operating room (OR) is rapidly contaminated by medical instruments and the surgical staff [10, 11]. Therefore, air quality control in the OR with a ventilation system is especially important to prevent SSIs.

Ventilation systems, particularly the use of a high efficiency particulate air (HEPA) filter, are widely used for air purification in clean ORs [12]. Ventilation system are generally composed of a HEPA filter and a diffuser attached to the ceiling centrally located above the operating table to allow the flow of clean air directly into the OR and displacement of contaminated air. Other ventilation systems utilize a diffuser that mixes clean air with the remnant contaminated air present in the OR. However, continuous displacement of contaminated air is key to minimize the abundance of airborne microorganisms and particles [12–14].

The first ventilation system used in China was installed in the OR of a Heilongjiang hospital in 1980, which was followed by the installation of 13 systems in Shenyang Military Area Command General Hospital in 1982 [15]. Since then, ventilation systems have been installed in most surgical centers in China to lower the risks of SSIs. Ventilation systems for ORs use state-of-the-art engineering technologies, thus continuous maintenance is particularly important for functional operation [16].

Relatively few studies have investigated compliance with air quality standards and management of ORs [17–19], and none, to the best of our knowledge, have identified factors associated with the management of air quality in clean ORs in China. Therefore, the aim of this study was to survey the usage, maintenance, and testing of ventilation systems in clean ORs among hospitals in China with the use of an online questionnaire.

## 2. Materials and Methods

### 2.1. Questionnaire Design and Online Survey

The questionnaire was divided into two parts: (1) basic information (type, level, and number of beds) and (2) usage and management (number of ORs, usage time, type of maintenance, test frequency, compliance with current standards, and comfort of the surgical staff). An electronic questionnaire was developed and data were collected using the Wenjuanxing™ platform (https://www.wjx.cn/). An online survey of medical institutions was conducted between August 5 and September 5, 2018 via the WeChat account of the Shanghai International Forum for Infection Control and Prevention. Participation in the survey was voluntary.

### 2.2. Standards for Maintenance of ORs in China

In accordance with the standards developed by the government of China (GB 50333: Architectural Technical Code for Hospital Clean Operating Departments), clean ORs were classified as one of the four grades based on the average concentration of airborne bacteria (colony-forming unit, CFU) as follows: grades I–III were defined as the presence of air diffusers installed on the ceiling of the OR and centralized located above the operating table with clean air directly supplied to the operating zone and surrounding areas, while grade IV was defined as the presence of air diffusers located on the ceiling with clean air diluting the contaminated air.

The average concentration of bacteria in ORs was classified as grade I (≤0.4 CFU/30 min (Petri dish diameter, 90 mm) or ≤10 CFU/m^3^), grade II (≤1.5 CFU/30 min (Petri dish diameter, 90 mm) or ≤50 CFU/m^3^), grade III (≤4 CFU/30 min (Petri dish diameter, 90 mm) or ≤150 CFU/m^3^, or grade IV (≤6 CFU/30 min (Petri dish diameter, 90 mm)). For each grade I OR, airflow was uniformly maintained at a rate of 0.20–0.25 m/s at 1.2 m above the floor. The minimum air changes per hour (ACH) for grade II, III, and IV ORs were 24, 18, and 12, respectively. Besides the airflow rate and ACH, other main technical parameters included were (1) positive pressure (vs. adjacent environment); (2) room temperature, 21–25°C; (3) relative humidity, 30%–60%; and (4) noise (grade I, ≤ 51 dB; grades II–IV, ≤V49 dB).

### 2.3. Statistical Analyses

Data were collected in an Excel file. Categorical variables were compared using the chi-square or Fisher's exact test. For convenience of analysis, continuous variables (number of beds, number of ORs, and usage time) were converted to ordered categorical variables. Maintenance of the ORs was performed in accordance with the GB 50333 standards and quantified based on the compliance rate. Univariate and multivariate logistic regression analyses were used to identify factors associated with the cleanliness of the ORs. Multivariate analyses were adjusted for the type of OR, hospital level, number of beds, and number of ORs. A probability (*p*) value of <0.05 was considered statistically significant. All data analyses were conducted using IBM SPSS Statistics for Windows, version 23.0. (IBM Corporation, Armonk, NY, USA).

## 3. Results

### 3.1. Basic Information of the Participating Hospitals

In total, 1318 responses to the questionnaires were received, of which 10 were incomplete, thus 1,308 completed questionnaires were included for analysis. Overall, 972 (74.31%) of the 1,308 ORs complied with the GB 50333 standards and 336 (25.69%) did not. Other information about the clean ORs is shown in Table 1.

### 3.2. Univariate Analysis of Factors Influencing Compliance with the GB 50333 Standards

Univariate analysis showed that two factors (i.e., maintenance mode and test frequency) were associated with compliance with the GB 50333 standards. Maintenance mode of “professional” was superior to “outsource or no” maintenance (*p* < 0.0001). Test frequency of “more than once a year” received a higher score than “occasionally or no” (*p* < 0.05). However, the type of OR, hospital level, number of beds, number of ORs, and usage time were not significantly associated with compliance with the GB 50333 standards (*p* > 0.05; Table 1).

### 3.3. Multivariate Analysis of Factors Influencing Compliance with the GB 50333 Standards

Multivariate analysis showed that factors influencing compliance with the GB 50333 standards included tertiary hospital level (odds ratio = 0.706, 95% confidence interval (CI) = 0.522–0.955, and *β* = −0.348), number of beds ≤1,000 (odds ratio = 0.696, 95% CI = 0.533–0.908, and *β* = −0.363), and professional maintenance (odds ratio = 0.511, 95% CI = 0.367–0.711, and *β* = −0.672). The type of OR (specialized vs. general), number of ORs, usage time, and test frequency had no significant influence on compliance with the GB 50333 standards (*p* > 0.05; Table 2).

### 3.4. Comfort of Healthcare Workers in ORs

In this study, the comfort of healthcare workers in ORs was investigated. Of 1308 respondents, 604 (46.17%) reported uncomfortable working conditions in ORs, mostly due to problems with humidity. Overall, there was a significant difference in the comfort of healthcare workers in ORs that complied with the GB 50333 standards vs. those that did not (39.92% [388/972] vs. 64.28% [216/336], respectively, *p* < 0.0001).

## 4. Discussion

The cleanliness of ORs has been correlated to the incidence of SSIs worldwide. However, the use of laminar (unidirectional) airflow (LAF) systems to prevent SSIs by achieving a higher level of cleanliness remains controversial [20–22]. The results of our online survey found that 25.69% of hospitals in China failed to comply with the GB 50333 standards. Further analysis found that routine testing and professional maintenance of ORs were positively correlated with compliance with the GB 50333 standards.

The “Global Guidelines for the Prevention of Surgical-Site Infection” of the World Health Organization recommend routine maintenance of ventilation systems, including installation of new filters, to prevent SSIs [16]. The GB 50333 standards and the WS/T 368 standard “Management specification of air cleaning technique in hospitals” [23] advise frequent changes of air filters, monitoring of the clean OR at least once per year, and a dedicated person responsible for clean OR maintenance. A prior study found that aerosols carrying *Mycobacterium chimaera* can penetrate laminar airflow and result in patient infections [24], demonstrating that the cleanliness of the air purification system in the OR is related to the incidence of SSIs.

In this study, 25.7% of the surveyed ORs failed to comply with the GB 50333 standards, similar to the rate of 20.0% reported in previous studies of clean ORs in China [25–27]. A study of 175 operating theatres under “at-rest” conditions and an “in operation” state, based on strict airborne microbial limits described in the Good Manufacturing Practice guidelines of the European Medicines Agency, found that the noncompliance rate with the Partial Unidirectional Airflow guidelines of the International Organization for Standardization (ISO) classes 5 and 7 was 10.8% and 1.8%, respectively, while the noncompliance rate of mixing airflow described in ISO 7 Types C and D was 20.3% and 10.1%, respectively [17]. A study conducted in Italy found that the airborne microbial load under “operational conditions” was higher than the reference value (>180 CFU/m^3^) in 13.03% of the tested ORs, while under “at-rest” conditions, 12.38% did not conform to the reference value (35 CFU/m^3^) [18]. The differences in noncompliance rates between the present and prior studies of ORs are due to differences in standards and evaluation items. In China, ORs are regularly monitored for compliance with the GB 50333 standards, which includes measuring microbe concentrations, cleanliness, ACH, pressure, temperature, humidity, and noise.

In the present study, routine testing and professional maintenance had the greatest influence the clean ORs operation, consistent with the guidelines of the World Health Organization and the GB 50333 standards [12, 16, 23]. A previous study reported that continuous maintenance of LAF and other technical systems was crucial because even minor failures of complex systems can have detrimental effects on air quality and patient safety [28]. Another study found that monitoring of microbes is useful to assess contamination of operating theatres and improve air quality [29]. Environmental factors in the clean OR, such as temperature, humidity, and fresh air supply, may not directly impact air quality but are equally important to maintain a comfortable working environment for healthcare workers. In this investigation, the most common complaint of healthcare workers was working under humid conditions, which was reported at a significantly higher rate among those in noncompliant ORs. A previous study reported that negative perceptions of task demands and distractions increased among surgical trainees in response to warmer temperatures [30].

Maintenance costs of clean ORs increase with the level of cleanliness. Clean ORs have recently become an important symbol of the modernization of hospitals in China, not only for tertiary hospitals, but secondary and lower level hospitals as well [13, 15]. Because relatively few high risk surgical procures are performed in secondary and lower level hospitals, the cost effectiveness of constructing clean ORs to prevent SSIs was investigated. The results showed no significant difference in the incidence of SSIs between ORs with state-of-the-art LAF systems as compared to conventional ORs [20–22]. However, the operation and maintenance of LAF systems in ORs are costly, averaging about 26,000 yuan (3,800 US dollars) per year [31]. Another study showed that the cost of an OR increased with the level of cleanliness, as the total maintenance cost of a grade I OR was more than 100,000 yuan (14,800 US dollars) per year [32]. Cost-effectiveness analyses conducted in other countries demonstrated that the use of a LAF system with a body exhaust suit resulted in higher costs but poorer health outcomes, thus these studies do not recommend the use of LAF systems [33, 34].

## 5. Conclusion

Our large-scale online survey of ORs in Chinese hospitals found that the maintenance was associated with clean OR operation. Hence, timely management of ORs should be prioritized to ensure cleanliness and comfort of healthcare workers and even minor failures of complex ventilation systems could result in detrimental effects in air quality and patient safety. In addition to ventilation systems, other air purification methods are recommended in the WS/T 368 standard to improve indoor air quality.

## Figures and Tables

**Table 1:** Univariate analysis of factors influencing compliance with the GB 50333 standards.

Influencing factors		Sample number	Noncompliance with the GB 50333 standards		*χ* ^2^	*p*
			Number, n	Rate, %		
Type of OR	Clean OR	966	243	25.2	0.549	0.459
	Clean OR and general OR	342	93	27.2		

Hospital level	Tertiary	677	164	24.2	1.752	0.416
	Secondary	594	163	27.4		
	Lower than secondary	37	9	24.3		

Number of beds	<500	453	111	24.5	2.574	0.276
	500–1,000	498	122	24.5		
	>1,000	357	103	28.9		

Number of ORs	<5	291	79	27.1	0.636	0.888
	5–9	432	106	24.6		
	10–15	287	75	26.1		
	>15	299	76	25.4		

Usage time (year)	≤5	464	114	24.6	0.472	0.492
	>5	844	222	26.3		

Maintenance mode	Professional	1,269	314	24.7	19.876	<0.0001^*∗*^
	Outsource or no	39	22	56.4		

Test frequency	More than once a year	1,117	274	24.5	5.374	0.020^*∗*^
	Occasionally or no	191	62	32.5		

^*∗*^Significance at *p* < 0.05.

**Table 2:** Multivariate analysis of factors influencing compliance with the GB 50333 standards.

Influencing factors	*β*	Standard error	Wald statistic	Odds ratio	95% CI	*p*
Type of OR	−0.033	0.151	0.047	0.968	0.719–1.302	0.829
Hospital level	−0.348	0.154	5.084	0.706	0.522–0.955	0.024^*∗*^
Number of beds	−0.363	0.136	7.118	0.696	0.533–0.908	0.008^*∗*^
Number of ORs	0.065	0.093	0.482	1.067	0.889–1.281	0.488
Usage time (year)	−0.080	0.148	0.318	0.923	0.699–1.219	0.573
Maintenance mode	−0.672	0.169	15.722	0.511	0.367–0.711	<0.0001^*∗*^
Test frequency	−0.152	0.087	3.028	0.859	0.724–1.019	0.082

^*∗*^Significance at *p* < 0.05.

## Data Availability

The data used to support the findings of this study are available upon request to the author.
